# Children's Neurological Status Epilepticus and Poor Prognostic Factors through Electroencephalogram Image under Composite Domain Analysis Algorithm

**DOI:** 10.1155/2021/8201363

**Published:** 2021-11-25

**Authors:** Runhan Zhang, Chao Gao, Junting Liu, Manting Zhao, Yongli Wu

**Affiliations:** Department of Child Healthcare, Cangzhou Central Hospital, Cangzhou 061000, Hebei, China

## Abstract

This study aimed to analyze the application of composite domain analysis algorithm for electroencephalogram (EEG) images of children with epilepsy and to investigate the risk factors related to poor prognosis. 70 children with neurological epilepsy admitted to the hospital were selected as the research objects. Besides, the EEG of the children during the intermittent and seizure phases of epilepsy were collected, so as to establish a composite domain analysis algorithm model. Then, the model was applied in EEG analysis. The clinical disease type and prognosis of children were statistically analyzed, and the risk factors that affected the prognosis of children were investigated. The results showed that the EEG signal values of the detail coefficients (d51 and d52) and the approximate coefficient (c5) during the epileptic seizure period were higher markedly than the signal values of the epileptic intermittent period; the EEG signal of the epileptic intermittent period was a transient waveform, which appeared as sharp waves or spikes. The EEG signal of epileptic seizures was continuous, with a composite waveform of sharp waves and spikes, and the change amplitude of the wavelet envelope spectrum during epileptic seizures was also higher hugely than that of intermittent epilepsy. The accurate identification rate, specificity, and sensitivity of EEG analysis with the composite domain algorithm were higher than those without the algorithm. Among the five types of epileptic seizures in children, the proportion of systemic tonic-clonic status was the largest, and the proportion of myoclonic status was equal to that of complex partial epileptic status, both of which were relatively small. The proportion of children with a better prognosis was 75.71% (53/70), which was higher than those with a poor prognosis 24.29% (17/70). Abnormal imaging examination (odds ratio (OR) = 3.823 and 95% confidence interval (CI) = 1.643–8.897); seizure duration greater than 1 hour (OR = 1.855 and 95% CI = 1.076–3.199); C-reactive protein (CRP) (OR = 5.089 and 95% CI = 1.507–17.187); and abnormal blood glucose (OR = 3.077, 95%CI = 1.640–5.773) were all independent risk factors for poor prognosis (all *P* < 0.05). The composite domain analysis algorithm was helpful for clinicians to find the difference in the EEG signals between the epileptic seizure period and the epileptic intermittent period in a short time, thereby improving the doctor's analysis of the results, which could reflect its marked superiority. In addition, abnormal imaging examinations, convulsion duration greater than 1 hour, CRP, and abnormal blood glucose were independent risk factors for poor prognosis in children. Therefore, the invasion of related risk factors could be reduced clinically by prognostic review with medical advice, attention to food safety and hygiene, and improvement of children's immunity.

## 1. Introduction

Children's neurological epilepsy is a common neurological syndrome caused by complex, recurrent, paroxysmal, and temporary brain dysfunction in children (0–18 years old). It is characterized by transient, rigid, paroxysmal, and repetitive central nervous system dysfunction. Its causes are mainly perinatal ischemia and hypoxia, cortical dysplasia, low-grade glioma, encephalitis, trauma, and so on, and it is a relatively common disease of children's nervous system [1]. Children can show sweating, convulsions, frequent convulsions, and even suffocation during the onset of the disease, which can easily cause loss of consciousness [2]. According to relevant epidemiological data, the prevalence of neurogenic epilepsy in children is about 6%, and there are at least 8.5 million children with epilepsy in China [3–5]. However, according to reports, the probability of intellectual impairment and structural abnormalities in epilepsy patients is about 20%–65%. Most of the patients have a chronic recurrent disease due to failure to detect and receive the appropriate treatment as early as possible and are accompanied by cognitive dysfunction, which seriously affects the healthy growth of children [6].

At present, the methods for detecting epilepsy in the clinic include computerized tomography (CT), magnetic resonance imaging (MRI), and EEG. What is more, EEG, the most commonly used technique in the clinic, uses electrical signals to record the activity of clusters of brain cells [7]. This examination technique appeared early in the 1970s, and a German professor named Hans Berger first recorded active currents from the human cerebral cortex in the 1990s. In 1935, researchers recorded 3 Hz pulses and ware complexes in the brains of epileptic patients such that slow comprehensive wave can further promote the application progress of EEG in clinical medicine [8]. Seizures will have physiological reactions similar to those of hysteria, syncope, migraine, and other diseases, which are easily confused [9]. Thus, it was necessary to use EEG inspection. According to relevant statistics, 83% of children with epilepsy have abnormal EEG. If proper EEG induction is performed, more patients will have abnormal EEG [10]. Epilepsy will not only damage the body of children but also leave children with sequelae and bring some social discrimination. Therefore, early detection and timely treatment are key to reducing children's neurological epileptic seizures [11].

The composite domain analysis algorithm was a multilead algorithm model that combined time-domain analysis, frequency-domain analysis, and time-frequency analysis. It can improve the efficiency of EEG data analysis and highlight its clinical application potential. In this study, 70 children with neurological epilepsy were selected, followed by EEG tracking. Then, the composite domain analysis algorithm was adopted to explore the clinical characteristics and prognostic factors of children with neurological epilepsy to provide a valuable reference for clinical treatment.

## 2. Materials and Methods

### 2.1. General Data

A total of 70 children with neurogenic epilepsy admitted to the hospital from June 2017 to March 2019 were selected as the research objects, including 38 male and 32 female children. Besides, they were from 1 month old to 17 years old, with an average age of 5.02 ± 1.24 years. There were 18 cases under 1 year, 20 cases between 1 and 3 years, 5 cases between 3 and 6 years, and 27 cases between 6 and 17 years. Based on the cause of the children, 23 cases suffered from central nervous system infection, 18 cases had hypoxic-ischemic encephalopathy, 14 cases had intracranial hemorrhage, and 15 cases suffered from head trauma. The diagnostic criteria were referred to the relevant diagnostic criteria in the 2006 International Anti-Epilepsy League Epilepsy Guidelines [12]. The inclusion criteria were defined to include children patients who met the above diagnostic criteria, did not take relevant antiepileptic drugs 3 months before treatment, were not contraindicated with antiepileptic drugs, were not allergic to the relevant treatment and examination drugs used in the treatment or examination in this study, and knew and signed the informed consent (their family members were aware of this study and also signed the informed consent). The exclusion criteria were defined to include children patients who were combined with cognitive impairment; had poor compliance and were unable to cooperate with the researchers; were accompanied by congenital heart disease, meningitis, and cerebrovascular malformations; suffered from abnormal liver and kidney function or were in a stressful state, and switched to other antiepileptic drugs during this study.

### 2.2. Research Methods

#### 2.2.1. EEG Collection

Before the examination, the children needed to remove their hair and wash their scalp, which should be kept clean and dry. The 16-lead video EEG system produced by Siemens, Germany, was used for examination. The electrodes, 2 reference electrodes, and the anti-interference ground wire were placed in 19 recording electrodes according to the l0–20 system. The scalp resistance of each electrode should be lower than 4.5 kW, the amplitude was 100 uV/cm, the speed of paper skip was 11 mm/s, and there was the routine unipolar lead tracing and the routine flash stimulation test. The monitoring should be continued for 18 hours, and one complete sleep cycle should be recorded at least. Then, the method of continuous playback was employed to intercept the complete EEG during the awake, sleepy, and nonrapid eye movement (NREM) phases. The videos of EEG after 3 months and 6 months of treatment of all children were rechecked to observe the change of EEG discharge frequency.

#### 2.2.2. Composite Domain Analysis Algorithm Model

Based on the children's EEG data, an epileptic EEG signal analysis algorithm of wavelet envelope spectrum was designed under composite domain analysis to better record and analyze the children's EEG data, and the valuable information could be extracted as the basis of clinical treatment.

First, the double-density discrete wavelet transform function was established, and the specific equation was as follows:

(1) $$\begin{array}{c} W\left(i\right)=\sqrt{2}\sum_{n}l_{0}\left(n\right)W\left(2i-n\right), \end{array}$$

(2) $$\begin{array}{c} P\left(i\right)=\sqrt{2}\sum_{n}l_{1}\left(n\right)W\left(2i-n\right). \end{array}$$

*W*(*i*) represented the scale function, *l*_0_ expressed the low-pass filter, *l*_1_ stood for the high-pass filter, and *P*(*i*) meant the wavelet number. *ls*(*n*),  *s*=0,1,2 should meet the following reconstruction conditions, which were presented as follows:.

(3) $$\begin{array}{c} L_{0}\left(t\right)L_{0}\left(\frac{1}{t}\right)+L_{1}\left(t\right)L_{1}\left(\frac{1}{t}\right)+L_{2}\left(t\right)L_{2}\left(\frac{1}{t}\right)=2, \end{array}$$

(4) $$\begin{array}{c} L_{0}\left(t\right)L_{0}\left(-\frac{1}{t}\right)+L_{1}\left(t\right)L_{1}\left(-\frac{1}{t}\right)+L_{2}\left(t\right)L_{2}\left(-\frac{1}{t}\right)=2. \end{array}$$

Thus, the following equations could be obtained:

(5) $$\begin{array}{c} W_{r}=W\left(i-r\right), \end{array}$$

(6) $$\begin{array}{c} P_{1,z,r}\left(i\right)=P_{1}\left(2^{z}i-r\right), \end{array}$$

(7) $$\begin{array}{c} P_{2,z,r}\left(i\right)=P_{2}\left(2^{z}i-r\right). \end{array}$$

Among them, there was {*z*, *r* ∈ *a*, *z* ≥ 0}, so the signal to be processed *y*(*i*) could be expressed as follows:

(8) $$\begin{array}{c} y\left(i\right)=\sum_{r=-\infty }f\left(r\right)W_{r}\left(i\right)+\sum_{s=1}^{2}\sum_{z=0}^{\infty }\sum_{r=-\infty }^{\infty }q_{s}\left(z,r\right)P_{s,z,r}\left(i\right). \end{array}$$

In the following equations, *f* and *q* stood for the low-frequency coefficient and the high-frequency coefficient, respectively:

(9) $$\begin{array}{c} f\left(r\right)=\int v\left(i\right)W_{r}\left(i\right)qi, \end{array}$$

(10) $$\begin{array}{c} q_{s}\left(z,r\right)=\int v\left(i\right)P_{s,r,z}\left(i\right)qi,\;s=1,2. \end{array}$$

Envelope spectrum analysis, also known as envelope demodulation analysis, is a very effective method for detecting periodic effects of signals, which is extensively used in mechanical fault diagnosis. In order to obtain a clearer and smoother envelope curve, the Hilbert transform formula was required as follows:

(11) $$\begin{array}{c} \bar{y}\left(i\right)=y\left(i\right)*\frac{1}{\Pi \Gamma }\\ =\frac{1}{\Pi }\int_{-\infty }^{\infty }\frac{y\left(\Gamma \right)}{i-\Gamma }a\Gamma . \end{array}$$

*y*(*i*) indicated the continuous-time signal, and Γ represented the transformation parameter. Moreover, an analytical signal was constructed by $\bar{y}\left(i\right)$ and *y*(*i*) in the above equation, as follows:

(12) $$\begin{array}{c} F\left(i\right)=y\left(i\right)+z\bar{y}\left(i\right). \end{array}$$

Then, the amplitude function could be obtained by taking the modulus value of *F*(*i*), which was expressed as follows:

(13) $$\begin{array}{c} O\left(i\right)=\left\lfloor F\left(i\right)\right\rfloor =\sqrt{{\left[y\left(i\right)\right]}^{2}+{\left[\bar{y}\left(i\right)\right]}^{2}}. \end{array}$$

The two were combined to analyze the wavelet envelope spectrum of epileptic brain signals, to effectively demodulate the low-frequency signal of each subband from the high-frequency signal in the wavelet domain.

#### 2.2.3. Algorithm Index

The commonly used indexes to evaluate the accuracy of the algorithm are accuracy (Acc), sensitivity (Sen), and specificity (Spe):

(14) $$\begin{array}{c} \text{Acc}=\frac{\text{TP}＋\text{TN}}{\text{TP}＋\text{TN}＋\text{FP}＋\text{FN}}\times 100\%,\\ \text{Sen}=\frac{\text{TP}}{\text{TP}＋\text{FN}}\times 100\%,\\ \text{Spe}=\frac{\text{TN}}{\text{TN}＋\text{FP}}\times 100\%. \end{array}$$

TP is the amount of positive data predicted as positive data, TV is the amount of negative data predicted as negative data, FP is the amount of negative data predicted as positive data, and FN is the amount of positive data predicted as negative data.

The double-density discrete wavelet transform decomposition coefficients and the corresponding coefficient envelope spectrum of the EEG signals in children patients were recorded during the intermittent and seizure periods of epilepsy. Since frequency components higher than 70 Hz lacked application value in research and analysis, the Butterworth low-pass filter was adopted to filter EEG signals to remove high-frequency interference. The EEG signals could be decomposed into several different frequency segments by using the compound domain analysis algorithm. These segments could not only separate the mutation signals of the EEG signals but also retain the time information of each segment, which can provide reference materials for the follow-up research. The wavelet envelope spectrum obtained in this study contained not only time-frequency information but also frequency-modulation and amplitude-modulation information, which better revealed the frequency and variation law of the mutation signal in the time-frequency domain. Moreover, the application of dual-density discrete wavelet transform also increased the ability to capture the signal details.

#### 2.2.4. Simulation Algorithm Flow

First, the epileptic EEG signal is processed, and the processing flow is shown in Figure 1.

Epilepsy EEG detection can be formalized as EEG signal classification. The classifiers used in this study are SVM, KNN, LDA, and DT. The four classifiers are introduced as follows.

  SVM: Map the data to a higher dimensional feature space, and then determine a hyperplane in this projection space to maximize the classification interval.
  KNN: The test sample category is determined based on the category of the *K* samples closest to it in the feature space; that is, the sample category belongs to most of the *k* nearest neighbor samples. The number of nearest neighbors *K* is the only parameter in the KNN model. If *k* = 1, the test sample category will be marked as the nearest neighbor sample category.
  LDA: It is a classical linear learning method, which projects historical data onto a straight line. After projection, it ensures that the distance between similar data is as close as possible and the distance between different types of data is as far as possible.
  DT: It is a nonparametric classifier, which derives decision rules according to the characteristics of training data. Its structure is similar to the flow chart, which is a directed tree composed of root nodes, internal nodes, and leaf nodes. Branching starts from the root node, where each internal node represents the test of a certain attribute of the data, and each leaf node represents the class or its distribution. Once the decision rules are generated and the tree structure is formed, the test data can be input into the tree and divided into different categories.

### 2.3. Statistical Processing

The collected data were sorted, summarized, and analyzed by SPSS 23.0. Measurement data were expressed as mean ± standard deviation (±*s*), and single sample data were represented by *t* test. In addition, *P* < 0.05 indicated that the difference was statistically substantial.

## 3. Results

### 3.1. Double-Density Discrete Wavelet Transform Decomposition Coefficients of EEG Signals and the Corresponding Coefficient Envelope Spectrum

Figures 2 and 3 show that the EEG signal values of the detail coefficients (d51 and d52) and the approximate coefficient (c5) of the epileptic period rose obviously in contrast to the signal values of the epileptic intermittent period. The interphase EEG signal was a transient waveform, which appeared as sharp waves. Besides, the EEG signal of epileptic seizures was continuous, with a composite waveform of sharp waves and spikes, and the change amplitude of the wavelet envelope spectrum in the seizure period was also greatly higher than that in the epileptic intermittent period.

### 3.2. Recognition Performance of the Composite Domain Analysis Algorithm

Figure 4 indicates that the correct recognition rate, specificity, and sensitivity of EEG analysis after using the algorithm were greater than the analysis value without using the algorithm, and the difference was statistically remarkable (^*∗*^*P* < 0.05).

### 3.3. Statistics of Types of Epileptic Seizures in Children

Among the five types of epileptic seizures in children, the proportion of systemic tonic-clonic status was the largest, the proportion of myoclonic status and complex partial status of epileptic status was equal to each other, and the difference was statistically obvious after comparison (^*∗*^*P* < 0.05) (Figure 5).

### 3.4. The Prognosis of all the Child Patients

Figure 6 reveals that the proportion of children with a good prognosis was 75.71% (53/70), which was higher than that of patients with a poor prognosis 24.29% (17/70), with a statistically marked difference (^*∗*^*P* < 0.05).

### 3.5. Single-Factor Analysis on the Prognosis of Children Patients

The single factor analysis showed that the proportion of imaging examination, convulsion duration, CRP, and blood glucose in children with good prognosis was statistically significant compared with the proportion of children with poor prognosis (*P* < 0.05), as shown in Table 1.

### 3.6. Multiple-Factor Analysis and Logistic Multiple-Factor Regression Analysis on Middle-Aged and Elderly Bronchial Asthma

The independent risk factors for poor prognosis in children included abnormal imaging examination, convulsion duration greater than 1 hour, CRP, and abnormal blood glucose (Table 2).

### 3.7. Comparison of EEG and Discharge Index in Children with Epilepsy before and after Treatment

The EEG discharge index of 70 children with epilepsy was 62.8 ± 12.567 before treatment and decreased significantly after treatment. There was a significant difference before and after treatment, *t* *=* 5.766, *P*=0.000 (^*∗*^*P* < 0.005). Figures 7 and 8 and Table 3 show the details.

## 4. Discussion

The clinical pathogenesis of epilepsy is relatively complicated, and a clear conclusion has not yet been obtained. Some studies believe that the disease is mainly caused by neurotoxicity, which leads to disorders of intracellular energy, thereby triggering the functions of breathing, liver, and kidney innervated by nerves. Obstacles cause the patients to have cognitive, behavioral, and local neurological deficits, which reduce the quality of life of the children and shorten the survival time of the child patients [13, 14]. Special examinations for children in the clinic include EEG and MRI, and EEG is critical evidence for the diagnosis of epilepsy. Therefore, most clinical doctors recommend that children's family members receive this examination, and the examination process will not make the child patient feel pain. Moreover, the clinical use rate is relatively high [15–17].

In order to improve the accuracy of the EEG examination results, the composite domain analysis algorithm was adopted in this study, the algorithm idea of wavelet envelope analysis was introduced into the field of epilepsy identification to reduce the influence of excessive fluctuation between single recognition data when the EEG signal analysis algorithm processed fixed classification tasks. Through systematic analysis of formic acid, the results of this study found that the interphase signal was a transient waveform, manifested as sharp waves or spikes, and the EEG signal of epileptic seizures is continuous, with a composite waveform consisting of sharp waves and spikes. Besides, the latter was brain waves to move more than the former, indicating that brain activity was relatively active in children with epilepsy. However, there were still differences between the intermittent EEG of epilepsy and the normal EEG because the intermittent EEG signal of epilepsy and the EEG signal of epilepsy were abnormal EEG. In this study, algorithm analysis was used, so that persevering clinicians could quickly differentiate and draw conclusions, which shortened the time of clinical diagnosis and promoted the treatment efficiency.

In this study, the clinical data and prognosis of the children were also analyzed. It was found that the generalized tonic-clonic status accounted for the largest proportion among the five types of epileptic seizures in children. Myoclonic status and complex partial status epilepticus accounted for the same proportion, and both had a smaller proportion. Furthermore, the proportion of children with a good prognosis was 75.71% (53/70), higher than that of patients with a poor prognosis (24.29%) (17/70). Statistical analysis of factors affecting the prognosis revealed that abnormal imaging examination, convulsion duration >1 hour, CRP, and abnormal blood glucose were all independent risk factors for poor prognosis in children patients.

According to a study by Hamano et al. [18], children with epilepsy with abnormal brain CT had a higher risk of poor prognosis, which corresponded to the results of this study. It might be because epilepsy was in a dynamic and constantly changing development process, so abnormalities occurred in daily cranial imaging examinations. According to the results of neuropathological studies, the continuous point activity abnormality of the central nervous system might result in irreversible neuronal damage and even death [19]. Children with recurrent clinical manifestations such as vomiting, nausea, vertigo, limb pain, headache, and abdominal pain, especially school-age patients, should be questioned on medical history in detail. If necessary, the corresponding auxiliary examination should be given. On the basis of excluding common diseases such as pediatric surgery, the disease should be highly suspected. Children should be treated immediately after their diagnosis, followed up, and observed, with paying attention to the toxic and side effects of drugs. They should be given early intervention and treatment in time, and their dose should be mastered. Half an hour after the onset of epilepsy, the child patient had brain hypoxia and decreased metabolic rate, and more than 1 hour could lead to permanent and irreversible brain damage. Therefore, the duration of convulsions longer than 1 hour was also one of the risk factors affecting the prognosis of children. Seizures can trigger a rapid stress response in the body, which increases the possibility of infection. What is more, CRP abnormalities are more common in infections, such as bacterial meningitis, sepsis, and other related encephalopathy. At the same time, studies have pointed out that blood glucose levels are not normal. The prognosis of children within the range is poor, and previous studies have confirmed that hypoglycemia can lead to brain damage [20]. Some children with poor prognosis in this study also suffered from hypoglycemia. Relevant researchers have also found that hyperglycemia is associated with the poor prognosis of patients with epilepsy. Therefore, it is necessary to understand whether children have the above risk factors during treatment and to diagnose and treat them in time [21].

## 5. Conclusion

To sum up, the composite domain analysis algorithm was applied in this study to analyze the EEG images of 70 children with neurogenic epilepsy, suggesting the difference between the EEG signals in the epileptic intermittent period and the epileptic period, which improved the doctor's understanding of the results. It also reflected the significant superiority of the composite domain analysis algorithm. In this study, the influencing factors of the patient's poor prognosis were also analyzed and sorted out, indicating that abnormal imaging examination, convulsion duration >1 hour, CRP, and abnormal blood glucose were independent risk factors for the poor prognosis of children patients. Therefore, the invasion of related risk factors could be reduced clinically through the prognostic review with medical advice, attention to food safety and hygiene, and improvement of children's immunity. In addition, researchers should continue to investigate the risk factors of poor prognosis in children patients with epilepsy and introduce them into the preventive treatment process to enhance rapid recovery of children patients.

The shortcomings of this study are that the description of the EEG research process is simple, and no more in-depth analysis has been carried out. Therefore, further in-depth discussions are needed in future research to better provide a clinical reference.

## Figures and Tables

**Figure 1:** Algorithm flow of epileptic EEG signal analysis.

**Figure 2:** Double-density discrete wavelet transform decomposition coefficients of EEG signals during intermittent epilepsy and the corresponding coefficient envelope spectrum.

**Figure 3:** Double-density discrete wavelet transform decomposition coefficients of EEG signals during epileptic seizures and the corresponding coefficient envelope spectrum.

**Figure 4:** Recognition performance of the composite domain analysis algorithm (compared with EEG analysis using the algorithm, ^*∗*^*P* < 0.05).

**Figure 5:** Statistics of epileptic seizure types in children (^*∗*^*P* < 0.05).

**Figure 6:** Comparison of the prognosis of the children patients (^*∗*^*P* < 0.05).

**Figure 7:** EEG after three months of treatment.

**Figure 8:** EEG after six months of treatment.

**Table 1:** Single factor analysis on prognosis of children (cases (%)).

Relevant factors		Good prognosis (*n* = 53)	Poor prognosis (*n* = 17)	*P* value
Gender	Male	25 (47.17)	9 (52.94)	>0.05
	Female	28 (52.83)	8 (47.06)	

Age (years old)	<6 years old	32 (60.38)	11 (64.71)	>0.05
	≥6 years old	21 (39.62)	6 (35.29)	

Imaging examination	Abnormal	45 (84.91)	14 (82.35)	<0.05
	Normal	8 (15.09)	3 (17.65)	

Past medical history	Yes	17 (32.08)	5 (29.41)	>0.05
	No	36 (67.92)	12 (70.59)	

Duration of convulsion (hour)	<1 hour	45 (84.91)	15 (88.24)	<0.05
	>1 hour	8 (15.09)	2 (11.76)	

CRP (mg/dL)	Abnormal	46 (86.79)	11 (64.71)	<0.05
	Normal	7 (13.21)	6 (35.29)	

Blood glucose (mmol/L)	Normal	47 (88.68)	7 (41.18)	<0.05
	Abnormal	6 (11.32)	10 (58.82)	

**Table 2:** Multiple-factor analysis on affecting the prognosis of children patients.

Factors	*β*	SE	Wald *χ*^*2*^ value	*P*	OR	95% CI
Abnormal imaging examination	1.341	0.431	5.024	0.002	3.823	1.643–8.897
Convulsion duration >1 hour	0.618	0.278	4.048	0.026	1.855	1.076–3.199
CRP	1.627	0.621	7.055	0.009	5.089	1.507–17.187
Abnormal blood glucose	1.124	0.321	4.353	≤0.001	3.077	1.640–5.773

**Table 3:** Changes of the EEG discharge index before and after treatment in 70 cases of children with epilepsy.

	Before treatment	After treatment	*t*	*P*
Discharge index	62.8 + 12.567	＜50	5.766	0.000

## Data Availability

The data used to support the findings of this study are available from the corresponding author upon request.
